# Premature Ventricular Contraction Recognition Based on a Deep Learning Approach

**DOI:** 10.1155/2022/1450723

**Published:** 2022-03-26

**Authors:** Nazanin Tataei Sarshar, Mohammad Mirzaei

**Affiliations:** ^1^Department of Engineering, Islamic Azad University Tehran North Branch, Tehran, Iran; ^2^Department of Electrical and Computer Engineering, Islamic Azad University Tehran North Branch, Tehran, Iran

## Abstract

Electrocardiogram signal (ECG) is considered a significant biological signal employed to diagnose heart diseases. An ECG signal allows the demonstration of the cyclical contraction and relaxation of human heart muscles. This signal is a primary and noninvasive tool employed to recognize the actual life threat related to the heart. Abnormal ECG heartbeat and arrhythmia are the possible symptoms of severe heart diseases that can lead to death. Premature ventricular contraction (PVC) is one of the most common arrhythmias which begins from the lower chamber of the heart and can cause cardiac arrest, palpitation, and other symptoms affecting all activities of a patient. Nowadays, computer-assisted techniques reduce doctors' burden to assess heart arrhythmia and heart disease automatically. In this study, we propose a PVC recognition based on a deep learning approach using the MIT-BIH arrhythmia database. Firstly, 10 heartbeat and statistical features including three morphological features (RS amplitude, QR amplitude, and QRS width) and seven statistical features are computed for each signal. The extraction process of these features is conducted for 20 s of ECG data that create a feature vector. Next, these features are fed into a convolutional neural network (CNN) to find unique patterns and classify them more effectively. The obtained results prove that our pipeline improves the diagnosis performance more effectively.

## 1. Introduction

According to the World Health Organization, the main cause of death worldwide is cardiovascular diseases (CVD). An evaluation proved that 17.9 million people died from CVD in 2019, indicating 32 of all global deaths [1]. According to the report of the sudden cardiac death in 2006 and latest standard in the American Heart Association (AHA) on ventricular arrhythmias, the epidemiology of ventricular arrhythmias entails a series of clinical applications and risk factors. These arrhythmias vary from sustained ventricular tachycardia, ventricular tachycardia, and premature complexes in people without cardiac problems background or ventricular tachyarrhythmia which leads to a sudden death [2]. Electrocardiogram (ECG) is a graph that records the fluctuations in electrical activity and is the main tool for predicting heart diseases. This ECG signal is generated by each heart cycle of the heart and can be recorded from the surface of each individual's body. Each ECG entails abundant pathological information and basic functions of the heart [3, 4]. Hence, it is a vital means for the diagnosis and examination of numerous arrhythmias. It is also of great importance to the assessment of cardiac safety and the assessment of numerous treatment techniques [4, 5].

A heart regular activity condition is reflected by a normal heartbeat (NB). Premature ventricular contraction (PVC) is a kind of ECG arrhythmias that is recognized to demonstrate an anomaly in the regular cardiac rhythm. PVC is the most common and widespread arrhythmia in the clinic, and it characterizes the abnormal behaviour of signals generated by ECG. PVC generates some variations in the heart rate leading to disruption in the electric and mechanic heart activity because of these delayed contractions (premature) [6, 7]. It means that PVC can be considered a kind of arrhythmia caused by an ectopic cardiac pacemaker represented in the ventricle. On the ECG, these PVCs are represented by bizarrely shaped and premature QRS complexes that have a *T* wave larger than normal and are typically wider than 120 ms. At present, doctors and experts can only employ the existing medical technology for recognizing PVCs using their personal experience. So, these decisions may lead to the wrong diagnosis because of long hours of high-intensity work. The issue of PVC diagnosis due to its pattern is quite changeable and is a challenging task, even for the same patient. Recently, employing ECG-based computer-aided diagnosis (CAD) systems, assisting doctors in the interpretation of PVC can successfully progress the efficiency of diagnosis [8–10].

In the last few years, machine learning (ML) approaches have gained much interest for the analysis of medical signals and images [11–16]. Deep learning (DL) pipelines are kinds of ML and have reached better feature extraction and classification outcomes compared to the state-of-the-art performance in the different fields of computer vision tasks [17–19].

Casas et al. [7] tried to simplify the process of extracting key features and employed some simple Bayesian generative models for classifying the extracted features. They used three classifiers including quadratic discriminant analysis (QDA), Gaussian linear discriminant analysis (LDA), and Gaussian Naïve Bayes (GNB). Twenty seconds of succeeding ECG beats that were recognized by an expert were used in [20] to characterize a PVC episode. They explored 7 statistical features and 3 morphological features. Then, all extracted features were normalized and used as the input of a classifier. They used an artificial neural network (ANN) for classifying these features to classify them into PVC or non-PVC classes. Oliveira et al. [21] suggested some simplified features and explored from geometric figures constructed over QRS complexes. In the first step, they rescaled the input signal using a wavelet denoising approach. Next, the signal was divided into separate parts to extract a new set of geometrical features. Finally, these extracted features were classified using eight different classifiers. Zhao et al. [22] suggested an approach by combining the convolutional neural network (CNN) and modified frequency slice wavelet transform (MFSWT). Firstly, in each recording, the first 10s ECG waveforms were transformed into time-frequency images employing MFSWT (frequency range of 0–50 Hz). Next, using a CNN model with 25 layers, these images are classified. The proposed CNN model comprises five convolution layers (kernel size of 3×3), five maximum pooling layers, five ReLU layers, a flatten layer, five dropout layers, and two fully connected layers.

In this paper, to overcome the problem of the similarity between PVC and non-PVC heartbeats, a deep learning approach is suggested which is based on an attention mechanism. Our pipeline not only obtains a high rate of accuracy but also diminishes the computation time.

## 2. Material and Method

We divide this section into two subsections. Firstly, we describe the method of extracting features from an ECG signal. Then, the process of finding more informative features employing a CNN model is described.

### 2.1. Feature Extraction

Feature extraction is a core building block of every artificial intelligence system. The main goal of the extracting features can be considered as finding distinct patterns (the most informative and compacted set of features) to increase the performance of the whole system [18, 23]. Besides, feature extraction is utilized for extracting features from the original 1D or 2D signals to perform a reliable classification task. This exploring step is the most fundamental part of each biomedical signal processing system because the performance of a classifier might be degraded if the features are not chosen well [24–26]. So, in this study, we aim to extract some key features from a ECG signal.

An example of a normal ECG signal is demonstrated in Figure 1. A normal ECG signal entails of 6 waveform parts: *T*, U, *R*, S, P, and Q. The fragment from *Q* to S is demonstrated as the QRS complex [9, 21, 22]. It represents ventricular depolarization and contraction and is a key clinical feature. Also, the distance among two maximum points indicates the length of a heartbeat and is demonstrated as the RR interval [6, 27, 28].

Group features play a significant role in the recognition of the PVR. The heartbeat and statistical features can be applied directly to the sequential RR cycle parts, so they are good features for applying to a real-time recognition system [28, 29].

Normally, the shape and size of the QRS complex are changed using the PVC, so it can be observed that the amplitude of the normal QRS complex is highly varied by the PVC [9]. In this study, for each ECG segment, we generate 10 distinct features that include 3 morphological features (RS amplitude, QR amplitude, and QRS width) and 7 statistical features implied in Table 1. The extracted statistical features comprise of the mean and standard deviation of the RR fragment. Also, it should be noticed that the percentage of differences among the neighboring RR intervals is greater than 10 ms or 50 ms (pRR10 and pRR50) [30–32]. An explanation of the time-domain features is demonstrated in Table 1.

By employing the MIT-BIH arrhythmia database, 10 heartbeats and statistical features are computed for each signal. The extraction process of these features is conducted for 20 s of ECG data that create a feature vector. Moreover, each group of features is labeled as non-PVC or PVC. For instance, a feature vector for a 20-second period is considered the PVC if it includes 95% PVC data; otherwise, it is labeled a non-PVC. Also, using the min-max normalization approach, we can normalize these features to values between zero and one by (1) before applying them into the CNN model for classification [6, 30].

(1) $$\begin{array}{c} \text{NV }=\;\frac{FV-F\text{min}}{F\text{max}-F\text{min}}, \end{array}$$

where FV is the feature value, NV implies the normalized value of the feature, *F*max and *F*min are the maximum and minimum values of features, respectively.

### 2.2. Our Deep Learning Model

In this section, we clarify how the suggested convolutional neural network (CNN) is able to learn more informative and unique details from the extracted features. Convolutional neural networks (CNNs) are kinds of neural networks (NNs) in the machine learning (ML) fields that mimic the behaviour of a human brain. CNNs are implemented to learn the distinct pattern and relationship between the input and the output signals or images employing their biases and weights [28, 33]. The key parts of every CNN structure include (1) convolutional (Conv) layer, (2) pooling layer, and (3) fully connected (FC) layer [4, 34].

Each Conv layer is specified by its kernel biases and weights which are specified in the training procedure by an iterative update process. These Conv layers accept random values at the beginning of the process and then regulated by backpropagation strategy to minimize a cost function. All obtained biases and weights are fixed in the testing Step [35, 36].

CNNs work by passing data through some stack of neurons, which are created as a series of layers. Usually, a nonlinear activation function (or squashing function) is applied to the extracted feature maps produced by a convolution layer. This activation function is responsible for computing the weighted sum of inputs and biases and then activate a neuron. Some widely used activation functions are sigmoid, Tanh, and rectified linear activation function (ReLU) [37, 38]. In this study, the ReLU activation function is employed.

Pooling layers are employed for reducing the size of the extracted feature maps. Consequently, it diminishes the number of neurons that need to be learned and the amount of computation performed in the network. The pooling layer summarizes the features present in an area of the feature maps created by the former Conv layer. Some widely used pooling methods are max-pooling and mean-pooling. In this study, the max-pooling is employed. Fully connected layer (FC layer) is simply, a feed forward neural network. The FC layer forms one or more last few layers in the network. These layers accept the output of the final pooling or Conv layer, which is flattened before applying [13–39]. Our network is displayed in Figure 2.

As clearly demonstrated in Figure 2, our CNN model accepts 10 features extracted from the last step and comprises of two feature extracting routes which are concatenated before applying to the FC layer. In the upper rout, there are four convolutional layers in which the first three of them do not use the pooling layer. In other words, the size of the input feature maps that are fed and are extracted from the first convolutional layers are the same. The first three Conv layers are responsible for extracting low-level features and the last Conv layer is used for extracting high-level features. The kernel size in all convolution layers is 3 × 3. We applied the pooling layer after the fourth convolution layer to decrease the dimension of the extracted feature maps. The next feature extracting route only has two convolution layers in which only the last one applies to the pooling layer. Also, the first and second Conv layers are responsible for extracting low-level and high-level features, respectively. These two separate routes permit the network to learn more informative details about the signal. The parameters utilized for training our network are described in Table 2.

## 3. Experiments

### 3.1. Dataset and Implementation Details

In this study, the available public MIT-BIH arrhythmia database is employed for assessment of our strategy experimental data [41, 42]. This standard database is one of the popular and broadly utilized ECG databases in the world. The database includes an overall of 48 records, each covering two 360 Hz signals, each with a length of 650,000 samples and a duration of approximately 30 minutes. The 48 records enclosed 23 records which are randomly chosen from more than 4,000 Holter recordings and numbered from 100 to 124 (some numbers missing). The rest of 25 records which numbered from 200 to 234 (some missing numbers) are clinically noteworthy arrhythmias but are the records of uncommon. The MIT-BIH data entail of three sections: (1) the comment file [atr] that employs binary storage, (2) the data file [dat] that is stored in the 212 format, and (3) the header file [hea] that is stored in the ASCLL code.

By exploring the MIT-BIH arrhythmia database, it is clear that the numbers of 102, 104, 107, and 217 cover paced beats. According to the Association for the Advancement of Medical Instrumentation (AAMI), we discard 4 records and use the rest of 44 records as investigational data. Moreover, to compare with some other structures, all remaining 44 records are divided into two datasets Data1 and Data2. Data1 is employed for training; Data2 is employed for testing. More details about them are shown in Table 3. Each dataset entails 22 records from the ECG database. Using the AAMI standard, there are five kinds of heartbeats: *Q*, V, S, F, and N. Before applying data into the classifier, we mark V type as PVC type and remaining as non-PVC so that the dataset entails only non-PVC and PVC groups.

### 3.2. Assessment Metrics

In this part, the assessment of the method is clarified. The performance of the model is evaluated by considering four basic criteria: true negative (TN), false positive (FP), false negative (FN), and true positive (TP). By using these four criteria, all the other statistical criteria can be computed. In this study, the true negative implies that the PVC was not identified, and the arrhythmia was not presented, while the true positive implies that a PVC was recognized and the arrhythmia actually happened. Moreover, the false negative demonstrates that a PVC was not recognized, whereas the arrhythmia was observed. Lastly, the false positive illustrates that a PVC was recognized, but it actually did not happen. Precision or positive predictive value (PPV) demonstrates the probability of being true positive when the test is positive. Sensitivity (true positive rate or recall) implies the ability of recognizing positive cases; the result with higher sensitivity has fewer false negatives samples. The F-score (F-measure) is a measure of a model's accuracy on a dataset. These three criteria are computed as follows [16, 23, 26]:

(2) $$\begin{array}{c} \text{sensitivity or recall }=\;\frac{TP}{TP+FN}\;\times 100. \end{array}$$

(3) $$\begin{array}{c} \text{PPV or precision }=\frac{TP}{TP+FP}\times 100\%. \end{array}$$

(4) $$\begin{array}{c} F=\;\frac{2\times \text{precision}\times \text{ recall}}{\text{precision}+\text{ recall}}\;\times 100\%. \end{array}$$

### 3.3. Experimental Results and Discussion

The suggested technique is implemented in MATLAB with the MatConvNet toolbox [43] on a PC with a GTX-1080 GPU, core i7 3.2 GHz CPU, and 8G memory.  Table 4 exhibits the performance of our strategy for some records. In this study, we use QRS fragment analysis as an appropriate tool, contributing to the revealing of ventricular hypertrophy, heart arrhythmias, and other diseases [5]. We observed that PVC beats (abnormal beats) entail QRS patterns broader than normal beats. Also, their statistical features are meaningfully diverse that permits PVC beats to be recognized comparatively easily [3]. Many varieties of arrhythmia, chiefly tachycardia and bradycardia, lead to changing in statistical features [27]. Accordingly, heartbeat and statistical features can be extracted directly from the sequential QRS cycle items. So, we extracted 10 features for each ECG fragment that play a key role for a classification task. For instance, from record No. 119 that entails many PVC beats in Table 4, it is clear that no PVCs were missed, but two wrong (false) alarms are observed over the 30-minute classification.

The PPV, F-score, and sensitivity values employing all mentioned frameworks are described in Table 5. For each index in Table 5, the highest PPV, F-score, and sensitivity values are highlighted in bold. Notice that when using the Yu et al.'s approach [6], PPV was enhanced in comparison to other strategies, but the values of recall utilizing the approaches by Allami et al. [20] and Xie et al. [31] are still higher. Additionally, there is a minimum difference between the values of recall employing those by Yu et al. [6] and Xie et al. [31]. Pierleoni et al. [44] gained the worst outcomes for all three measures. There was a diminish chiefly in the positive class scores.

Moreover, it is clear that our approach and Allami et al.'s approach [20] are more stable than the Grad-CAM by Pierleoni et al. [44] and Xie et al. [31]. Meanwhile, Xie et al. [31] showed the same performance, getting only one more false negative and two more false positives. For Pierleoni et al. [44], all measures are less than the other approaches and it suffers from overfitting. The gap between the values of PPV by employing Yu et al. [6] and Allami et al.'s approaches [20] is not significant which is relatively smaller than this gap when using Xie et al. [31] and Pierleoni et al.'s approaches [44]. In ML techniques, how to design a suitable feature exploring technique is a challenge task and the classification performances are lower than the suggested pipeline. Moreover, our technique not only enhances the accuracy of traditional ML strategies but also is capable of automatically exploring and biasing key features of raw ECG signals.

## 4. Discussion and Conclusions

In this study, a novel premature ventricular contraction recognition based on a deep learning approach has implemented benefits from the characterization of an ECG signal. It means that each ECG signal has many informative and unique characteristics to aid our method efficiently even if dissimilar shapes are presented. We employed 10 distinct features that include 3 morphological features (RS amplitude, QR amplitude, and QRS width) and 7 statistical features which are able to highlight distinction between different parts of ECG signals. Moreover, we have employed a CNN structure for identifying more unique features that allows our pipeline to reach a higher classification performance. This approach leads to diminishing the false positive rate and increasing the true positive rate. Moreover, our technique not only enhances the accuracy of traditional ML strategies but also is capable of automatically exploring and biasing key features of raw ECG signals. We conducted comprehensive investigations, which demonstrate the effectiveness of our technique by the comparison with the state-of-the-art strategies [40].

## Figures and Tables

**Figure 1:** An example of a normal ECG signal [27].

**Figure 2:** The proposed CNN structure with two separate feature extracting routes.

**Table 1:** Explanation of statistical features.

Features	Explanation
SDSD	Standard deviation of dissimilarities among sequential RR intervals.
Ratio	Ratio=(maxRR −minRR)/*μ*rr
rMSSD	Square root of the mean of the squares of dissimilarities among neighboring RR intervals.
SDRR	Standard deviation of all RR intervals
pRR10	Percentage of dissimilarities among neighboring RR intervals that are greater than 10 ms.
pRR50	Percentage of dissimilarities among neighboring RR intervals that are greater than 50 ms.
MeanRR	Mean value of all RR intervals (*μ*)

**Table 2:** Parameters utilized to train our network.

Parameters	Value
Input features	10 × 1
Output classes	2
Learning rate	0.0001
Max epochs	40
Activation function	Softmax
Batch size	200
Optimizer	Adam
Learning rate drop factor	0.2

**Table 3:** Description of the dataset and partitioning of all signals.

Data	Signals	Used for train or test	PVC type (V)	Non-PVC type (non-*V*)	Total
Data2	100, 103, 105, 111, 113, 117, 121, 123, 200, 202, 210, 212, 213, 214, 219, 221, 222, 228, 231, 232, 233, 234	Test	3157	46539	49696
Data1	101, 106, 108, 109, 112, 114, 115, 116, 118, 119, 122, 124, 201, 203, 205, 207, 208, 209, 215, 220, 223, 230	Train	3648	47573	51221
DS1 + DS2	44 signals	-	6805	94112	100917

**Table 4:** The performance of our strategy for some records.

Record no.	PPV	Recall	F-score	Record no.	PPV	Recall	F-score
100	99.5	100	99.7	201	97.5	94.1	95.8
105	95.4	94.3	94.8	210	98.7	96.3	97.5
113	98.2	93.1	95.3	217	95.2	91.9	93.1
119	97.3	100	98.3	231	97.8	93.7	95.7

**Table 5:** Comparison between the suggested network and other baseline models on MIT-BIH arrhythmia database.

Method	PPV (mean)	Recall (mean)	F-score (mean)
Allami et al. [20]	97.8	98.7	98.2
Pierleoni et al. [44]	86	87	86.5
Xie et al. [31]	95.4	97.8	96.6
Yu et al. [6]	98.1	97.2	97.6
Our approach	98.6	99.2	98.9

## Data Availability

In this study, the available public MIT-BIH arrhythmia database is employed for assessment of our strategy experimental data.
